# Inhibition of the Receptor Tyrosine Kinase ROR1 by Anti-ROR1 Monoclonal Antibodies and siRNA Induced Apoptosis of Melanoma Cells

**DOI:** 10.1371/journal.pone.0061167

**Published:** 2013-04-08

**Authors:** Mohammad Hojjat-Farsangi, Fatemeh Ghaemimanesh, Amir Hossein Daneshmanesh, Ali-Ahmad Bayat, Jafar Mahmoudian, Mahmood Jeddi-Tehrani, Hodjatallah Rabbani, Hakan Mellstedt

**Affiliations:** 1 Department of Oncology-Pathology, Immune and Gene therapy Lab, Cancer Center Karolinska (CCK), Karolinska University Hospital Solna and Karolinska Institute, Stockholm, Sweden; 2 Department of Immunology, School of Medicine, Bushehr University of Medical Sciences, Bushehr, Iran; 3 Monoclonal Antibody Research Center, Avicenna Research Institute, ACECR, Tehran, Iran; Dana-Farber Cancer Institute, United States of America

## Abstract

The receptor tyrosine kinase (RTK) ROR1 is overexpressed and of importance for the survival of various malignancies, including lung adenocarcinoma, breast cancer and chronic lymphocytic leukemia (CLL). There is limited information however on ROR1 in melanoma. In the present study we analysed in seven melanoma cell lines ROR1 expression and phosphorylation as well as the effects of anti-ROR1 monoclonal antibodies (mAbs) and ROR1 suppressing siRNA on cell survival. ROR1 was overexpressed at the protein level to a varying degree and phosphorylated at tyrosine and serine residues. Three of our four self-produced anti-ROR1 mAbs (clones 3H9, 5F1 and 1A8) induced a significant direct apoptosis of the ESTDAB049, ESTDAB112, DFW and A375 cell lines as well as cell death in complement dependent cytotoxicity (CDC) and antibody dependent cellular cytotoxicity (ADCC). The ESTDAB081 and 094 cell lines respectively were resistant to direct apoptosis of the four anti-ROR1 mAbs alone but not in CDC or ADCC. ROR1 siRNA transfection induced downregulation of ROR1 expression both at mRNA and protein levels proceeded by apoptosis of the melanoma cells (ESTDAB049, ESTDAB112, DFW and A375) including ESTDAB081, which was resistant to the direct apoptotic effect of the mAbs. The results indicate that ROR1 may play a role in the survival of melanoma cells. The surface expression of ROR1 on melanoma cells may support the notion that ROR1 might be a suitable target for mAb therapy.

## Introduction

Melanoma is a skin cancer arising from melanocytes located in the epidermis. The incidence of melanoma is rapidly increasing. The frequency of melanoma is only 4% of all dermatological cancers but responsible for 80% of the mortality in skin cancer. Early detection and treatment may improve prognosis [1]. A series of melanoma-associated antigens (MAGE) has been identified on melanoma cells [2]–[4]. Large efforts have been done to use different MAGEs for immunotherapy of melanoma patients, but most clinical trials have failed [5].

Receptor tyrosine kinases (RTKs) are important structures involved in cell signaling, differentiation and proliferation of normal and malignant cells [6]. RTKs and their signaling pathways may contribute to the dysregulation of malignant cells, as self-sufficiency for growth factors, evasion from apoptosis, unlimited cell replication and metastasis [7]. The receptor tyrosine-kinase-like orphan receptor 1 (ROR1) is a member of the RTK families [8]–[11] and a highly conserved receptor with no clearly identified ligand/s [12]. Wnt5a has however been suggested as a candidate ligand for ROR1 [9], [13]–[14].

ROR1 is a transmembrane protein consisting of 937 amino acid residues with an extra and intracellular part. The extracellular part consists of 3 regions, including the Ig-like, cysteine rich (CRD) and kringle (KNG) domains. The CRD and KNG domains might be ligand binding sites [13], [15]. The intracellular part contains a tyrosine kinase domain that might be triggered to phosphorylation by other cytoplasmic signaling proteins [16]. ROR1 is expressed during the development of the nervous system and regulates survival and maintenance of neural progenitor cells in the brain [14]. It is also expressed in other organs during embryogenesis and of importance for the morphogenesis of several organs [12].

The role of ROR1 in various malignancies is not well understood. No mutations have been noted [17]. ROR1 is however considered to be a survival factor for various malignancies including chronic lymphocytic leukemia (CLL) [18], breast cancer [13] and lung adenocarcinoma [15]. ROR1 might be a promising antigen to be targeted. Anti-ROR1 monoclonal antibodies (mAbs) and ROR1 specific siRNAs have been shown to induce apoptosis and necrosis of malignant cells [16], [19]–[20].

In the current study, we analysed the expression and phosphorylation of ROR1 in a series of malignant melanoma cell lines using RT-PCR, immunocytofluorescence (IF), flow cytometry and western blot. The cytotoxic effects of anti-ROR1 mAbs were evaluated in the absence or presence of complement (complement dependent cytotoxicity) (CDC) or immune effector cells (antibody dependent cell-mediated cytotoxicity) (ADCC) and ROR1 siRNA was used for gene silencing.

## Materials and Methods

### Cell lines and controls

The melanoma cell lines ESTDAB049, 075, 081, 094 and 112 were obtained from the European Searchable Tumor Cell Line Data Base (ESTDAB project, contract no. QLRI-CT-2001- 01325) [21]. The DFW melanoma cell line was derived from a metastatic lesion from a patient at Radiumhemmet, Karolinska Hospital University Solna, Stockholm, Sweden [22]. A375 (melanoma cell line) and T47D (human ductal breast epithelial tumor cell line) were obtained from American Type Culture Collection (ATCC). After thawing, cells were grown in RPMI-1640 (Gibco, Life Technologies, Karlsruhe, Germany) containing 10% FCS (Gibco), 2% glutamine (Biochrom KG, Berlin, Germany) and 100 ug/ml penicillin/streptomycin (Biochrom KG) (complete medium) at 37°C in a humidified incubator with 5% CO_2_.

### Production of anti-ROR1 monoclonal antibodies

Mouse monoclonal antibodies against ROR1 were generated against the extracellular part of ROR1 as previously described [20]. Out of more than 20 clones, four clones including 1A8, 1E9, 5F1 and 3H9 (all of the IgG1 isotype) were selected. The characterization and specificity of the anti-ROR1 mAbs (Avicenna Research Center, Tehran, Iran) were checked by ELISA and after transfection of the HEK293 cell line with the extracellular domain of ROR1 in western blot as previously described [17].

### RNA preparation, cDNA synthesis and RT-PCR

Total RNA was purified from cells, using pure link RNA mini-kits (Ambion, Inc., Austin, Texas, USA). One ug of high quality RNA was reversely transcribed using a first strand cDNA synthesis kit (Fermentas, St. Leon-Rot, Germany) according to the manufacturer's instructions. PCR amplification was performed as previously described [23], using 150 ng of cDNA for PCR amplification. ROR1 specific primers, 5′-CTGCTGCCCAAGAAACAGAG-3′ (position 455–474) as the sense and 5′-CATAGTGAAGGCAGCTGTGATCT-3′ (position 977–999) as antisense primers, with a PCR product of 545 bp (reference: g.b. M97675) were used for ROR1 amplification [17]. Beta-actin was used as a control for cDNA quality and integrity (Sense primer: ATTAAGGAGAAGCTGTGCTACGTC, Anti-sense primer: ATGATGGAGTTGAAGGTAGTTTCG) [17].

### Immunocytofluorescence (IF)

Cells were grown on coverslips (Marienfeld GmbH & Co, Lauda-Königshofen, Germany) placed in 35-mm dishes in an incubator with humidified air and 5% CO_2_ at 37°C. After 24 h of incubation, medium was removed. Cells were dried at room temperature (RT) and fixed with cold neutral buffered formalin for 5 min. The slides were washed with tris-buffered saline (pH = 7.4), containing 0.1% Bovine Serum Albumin (TBS-BSA) and blocked with 5% sheep serum diluted in TBS-BSA for 30 min. Slides were then incubated with 5 ug/ml of ROR1 mAbs as well as with a non-relevant mAb (mouse IgG1 isotype) (eBioscience, Inc., San Diego, California, USA) for 1 h at RT. Following three washes, slides were incubated with FITC- conjugated sheep anti-mouse IgG (1∶100) (Avicenna Research Center) for 1 h. After three washes in TBS-BSA, the nuclei were counterstained with 1 ug/ml of 4′, 6-Diamidino-2-Phenylindole Dihydrochloride (DAPI) (Sigma-Aldrich Corp., Saint Louis, MO) for 5 min. Finally, cells were mounted in PBS-glycerol 50% and examined with a fluorescent microscope (Zeiss Axioplan2, Oberkochen, Germany).

### Flow cytometry analysis

Surface staining of cells was performed as previously described [24]. Briefly, 10^6^ cells were washed in PBS and suspended in 100 ul of FACS buffer (PBS, 0.1% sodium azide, and 0.5% BSA). Five ug/ml of the respective anti-ROR1 mAbs or one ug/ml of polyclonal goat anti-ROR1 antibody (R&D system, Minneapolis, MN, USA) was added to the cells and incubated at 4°C for 1 h. Cells were washed with FACS buffer and FITC conjugated sheep anti-mouse Ig or FITC conjugated rabbit anti-goat Ig (Dako, Glostrup, Denmark) (1∶100) were added and incubated at 4°C for 1 h. Finally, cells were washed with FACS buffer and fixed with 1% paraformaldehyde in PBS. A FACSCalibur flow cytometer (BD Bioscience, Mountain View, CA, USA) was used to analyse ROR1 expressing cells. 5×10^4^ events were counted. Cells were analyzed using the FlowJo software program (Tree Star Inc. Ashland OR, USA).

### Western blot analysis

10×10^6^ cells were lysed in 200 ul of lysis buffer [0.1% SDS, 1% Triton X-100, 50 mM Tris- HC1, pH 7.4, 150 mM NaCl, 5 mM EDTA, 1% protease inhibitor cocktail (Sigma-Aldrich) and phosphatase inhibitor (Roche, Stockholm, Sweden)] and incubated on ice for 30 min with 5 min interval and vortexed for 10 sec. Bicinchoninic acid (BCA) protein assay kit (Thermo Scientific, IL, USA) was used to measure the protein concentration according to the manufacturer's instructions. Ten ug of the cell lysate or immunoprecipitated ROR1 (using goat anti-ROR1 antibody) was run on 10% Bis-Tris SDS-PAGE gel at 120V/90mA for 2 h (IP-WB). After electrophoresis, proteins were transferred to PVDF membrane (Millipore Corporation, Bedford, MA, USA) and blocked overnight at 4°C with 5% nonfat dry milk (skim milk) or BSA in TBS containing 0.1% Tween 20 (TBS-T). Filters were incubated with anti-phospho-tyrosine (0.5 ug/ml) (PY99, Santa Cruz Biotechnology, Inc., CA, USA), anti-phospho-serine mAbs (clone 4A4) (0.5 ug/ml) (Millipore Corporation) or goat anti-ROR1 polyclonal antibody (R&D system) (0.2 ug/ml) for 1 h at RT. After washing with TBS-T, filters were incubated with peroxidase-conjugated rabbit anti-goat or rabbit anti-mouse immunoglobulin (Dako) for 1 h at RT followed by washings and developed using the advanced ECL chemiluminescence detection system (GE Healthcare, Uppsala, Sweden).

Cleaved PARP as well as caspase-8 and 9 and MCL-1 expression were analyzed using cell lysates from the apoptosis experiments (see below). Briefly, 10 ug of the protein lysate was run in western blot. Filters were incubated with rabbit anti-PARP, cleaved caspase-8 (p 43/41 and p18), cleaved caspase-9 (p37) and MCL-1 antibodies (Cell Signaling Technology, Danvers, MA, USA) respectively overnight at 4°C, and subsequently with a peroxidase-conjugated goat anti-rabbit antibody (Dako). Finally, blots were developed with a chemiluminescence detection system [20].

### Annexin-V/PI apoptosis assay

5×10^4^ cells/well were cultured in 6 replicates in 24 well plates. After 24 h, medium was replaced and cells were incubated with 5 ug/ml of the ROR1 mAbs in 1 ml of complete medium. Cells treated with a non-relevant isotype control mAb (mouse IgG1 isotype) (eBioscience) or 1 uM staurosporine (Sigma-Aldrich) were used as controls, respectively. After 24 h of incubation at 37°C in humidified air with 5% CO_2_, cells were collected (24 well plates were incubated on ice for 10 min and then cells were suspended by pipetting), washed twice with PBS and resuspended in 150 ul of binding buffer. Five ul of FITC-conjugated Annexin-V and PI (propidium Iodide) (BD Biosciences) was added to the cells, vortexed and incubated at RT in the dark for 10 min. Apoptosis was measured by flow cytometry (FACSCalibur, BD Biosciences). Cells were analyzed using the FlowJo software program.

### XTT cytotoxicity assay

XTT (2,3-bis-(2-methoxy-4-nitro-5-sulfophenyl)-2H-tetrazolium-5-carboxanilide) cytotoxicity assay was used as previously described [25]. Briefly, 10^4^ cells were incubated in 200 ul complete medium in 6 replicates using 96 well plates. After 24 h, medium was replaced and anti-ROR1 mAbs were added to the cells (5 ug/ml) as well as the non-relevant isotype control mAb (mouse IgG1 isotype). The T47D cell line treated with mAbs was used as a negative control [16]. Cells were incubated for 24 h with mAbs and 20 ul of XTT (5 mg/ml) (Sigma-Aldrich) in PBS was added after activation of XTT with PMS (N-methyl dibenzopyrazine methyl sulfate) (Sigma-Aldrich). Cells were incubated for further 2 h at RT. Optical density (OD) was measured at 450 nm. Cytotoxicity was calculated as follows: % cytotoxicity = (Test OD - background OD)/(positive control OD - background OD)×100. The positive control OD was defined as the value of untreated cells at time zero and background OD as the value of medium alone.

### CDC and ADCC assays

The effect of anti-ROR1 mAbs in CDC was evaluated as previously described [26]. Briefly, 5×10^4^ target cells were plated in V-bottomed microtiter plates (Nunc, Roskilde, Denmark) in 100 ul complete medium. Cells were incubated with 5 ug/ml of each of the anti-ROR1 mAb as well as with 5 ug/ml of the non-relevant isotype control mAb (mouse IgG1 isotype) for 30 min at RT followed by washings with RPMI-1640. Twenty percent fresh normal human serum (NHS) in 100 ul complete medium was added and cells incubated at 37°C in a humidified air with 5% CO_2_ for 2 h. Finally, cells were collected, washed twice with PBS and resuspended in 150 ul of Annexin-V/PI binding buffer. Five ul of PI was added to the cells, vortexed and incubated at RT in the dark for 10 min. The frequency of PI stained cells was measured by flow cytometry.

ADCC assay was performed as previously described [20]. Briefly, cells were labeled with 2.8 MBq sodium Cr51 (PerkinElmer Inc. Wellesley, MA, USA) for 3 h at 37°C. After 3 washes with RPMI-1640, 10^4^ cells in 100 ul medium were added to each round-bottomed microtiter well (Nunc) and natural killer (NK) cells enriched from healthy donors buffy coat [26] were added to yield target: effector cell ratios of 1∶25 and 1∶50 to a final volume of 200 ul containing 5 ug/ml of the anti-ROR1 mAbs or the non-relevant isotype control mAb (mouse IgG1 isotype). Each experiment was run in six wells. After 4 h at 37°C, the reaction was stopped by centrifugation. Cr51 release was measured by a gamma counter (Beckman Gamma 5500, Beckman Coulter, Fullerton, CA). The percentage of target cell lysis was calculated based on the following formula: % specific lysis = (experiment cpm- spontaneous cpm)/(maximum cpm-spontaneous cpm)×100. Maximum Cr51 release was determined by adding 1% of Triton X-100 to the target cells and spontaneous release was measured in the absence of antibodies and effector cells.

### ROR1 siRNA transfection

Downregulation of endogenous ROR1 mRNA was performed as previously described [19]. The siRNA sequences used to target 5′-ATGAACCAATGAATAACATC-3′ ROR1 mRNA with antisense 5′-GAUGUUAUUCAUUGGUUCAdTdT-3′ and sense 5′-UGAACCAAUGAAUAACAUCdTdT-3′ sequences. Control siRNA (MISSION siRNA Universal Negative Control; Sigma-Aldrich) was used as a negative control. Cells were harvested after 6, 12, 24 and 36 h of incubation for mRNA preparation, the Annexin-V/PI apoptosis assay and for western blot.

### Data analysis

Statistical analyses were performed using student's t-test and Mann–Whitney U test as appropriate. Analyses were conducted using the SPSS statistical package (SPSS, Chicago, IL). P-values less than 0.05 were considered to be significant.

## Results

ESTDAB (European Searchable Tumor Cell Line Database) contains more than 100 melanoma cell lines with defined HLA class I and II genotypes in the ESTDAB Melanoma Cell Bank (Tubingen, Germany). These cell lines also have been characterized for glycan composition in relation to clinical tumor progression [21], [27]–[29]. In the current study, we randomly selected five cell lines (049, 075, 081, 094 and 112) from this collection and two other melanoma cell lines (A375 and DFW).

### ROR1 expression and phosphorylation

The expression of ROR1 mRNA was determined by RT-PCR. ROR1 was expressed in all melanoma cells at the mRNA level but not in the T47D cell line. The protein expression of ROR1 was assessed by IF. All melanoma cell lines expressed the ROR1 molecule (anti-ROR1 mAb clone 3H9). Representative results for the ESTDAB112 cells are shown in Figure 1A. In IP-WB (immunoprecipitation followed by western blot), a 130 kDa band representing fully glycosylated ROR1 was detected using a goat anti-ROR1 polyclonal antibody for immunoprecipitation. This band could also be shown to be phosphorylated using anti-phospho-tyrosine and phospho-serine mAbs. No expression of ROR1 was seen in the T47D cell line [16] (Fig. 1B).

**Figure 1:** Protein expression of the receptor tyrosine kinase ROR1 in melanoma cell lines. Representative experiment (IF) showing the expression of ROR1 on the ESTDAB112 cell line using the anti-ROR1 (clone 3H9) mAb (40×). Nuclei were counterstained with DAPI (blue). A non-relevant isotype control mAb (mouse IgG1 isotype) was used as a negative control (A). Western blot analysis of ROR1 protein expression and phosphorylation in melanoma cells detected by a goat anti-ROR1 antibody, anti-p-tyrosine (PY99) and anti-p-serine (clone 4A4) mAbs (B). ROR1 protein was shown to be phosphorylated in all cell lines using immunoprecipitation of ROR1. A 130 kDa band corresponding to the fully glycosylated/phosphorylated ROR1 was observed. The T47D cell line was used as a ROR1 negative control [16].

ROR1 surface expression and intensity was also analysed by flow cytometry. All cell lines expressed ROR1 as detected by the four anti-ROR1 mAbs and a polyclonal goat anti-ROR1 antibody (Table 1). However it should be noted that a proportion (about 50%) of the melanoma cells did not express ROR1.

**Table 1:** Frequency of ROR1 positive melanoma cells.

ROR1 mAb			ESTDAB					
	049	075	081	094	112	DFW	A375	T47D
**1A8**	60 (17.1)	52.5 (16)	60 (60.3)	59.1 (54.5)	52.3 (19.7)	59.4 (52.1)	57.9 (36.7)	5 (3)
**1E9**	64.3 (27)	53.6 (14)	63.5 (38.6)	75.2 (113)	58.6 (23)	65 (74)	44 (12.5)	11 (4)
**5F1**	68.9 (29.3)	59.3 (22.3)	62.5 (40.4)	70.9 (46.6)	56.8 (15.8)	68.3 (47.5)	71.3 (86.4)	9 (5)
**3H9**	78.1 (99.6)	58.4 (22.2)	70 (74.2)	70.4 (46.7)	63.7 (24.1)	62.4 (85.7)	58.7 (56.9)	5 (3)

Frequency (%) of ROR1 positive cell lines and Geometric Mean Fluorescence Intensity, stained by 4 anti-ROR1 mAbs in flow cytometry.

### Induction of apoptosis by anti-ROR1 mAbs

Induction of apoptosis by the anti-ROR1 mAbs in the absence of complement or effector cells was analysed after 24 h incubation (Fig. 2). The frequency of apoptotic/necrotic cells (lower right, upper left and right quadrants) induced by a non-relevant isotype control mAb (mouse IgG1 isotype) was deducted from the frequency of cells treated with the anti-ROR1 mAbs. Anti-ROR1 mAbs alone induced apoptosis of melanoma cells varying between 4% and 54% as determined by Annexin-V/PI staining (Fig. 2A) and the XTT assay (Fig. 2B). Representative experiments are shown in Figure 2C. Different anti-ROR1 mAbs had various effects on the individual cell lines. The anti-ROR1 mAb clones 5F1, 3H9 and 1A8 were the most effective using ESTDAB049, ESTDAB112, DFW and A375 cell lines, while anti-ROR1 mAb clone 1E9 was the most effective using ESTDAB075 cells. ESTDAB081 and 094 cell lines were resistant to the direct cytotoxic effects of the anti-ROR1 mAbs. The frequency of ROR1 positive cells did not differ significantly comparing the various melanoma cell lines. No effect on apoptosis of the non-relevant isotype control mAb (mouse IgG1 isotype) was observed. The anti-ROR1 mAbs did not induce apoptosis of the ROR1 negative cell line T47D.

**Figure 2:** Induction of apoptosis in melanoma cells using anti-ROR1 mAbs. Frequency (%) of apoptotic/necrotic cells in Annexin-V^+^/PI^+^ (A) and XTT cytotoxicity assay (B) induced by anti-ROR1 mAbs in the absence of complement or immune effector cells [anti-ROR1 mAb clones 1A8 (□), 1E9 () and 5F1 ()3H9 (▪)]. Dot plot diagrams of apoptosis induced by anti-ROR1 mAbs (clones 1A8 and 3H9) in melanoma cells and ROR1 negative cell line T47D (Annexin-V/PI) (C). Western blot for cleaved PARP, caspase 8, 9 and MCL-1 expression in apoptotic ESTDAB049 and ESTDAB112 cells induced by the anti-ROR1 mAb clone 5F1 (D). (−) cells treated with a non-relevant isotype control mAb (mouse IgG1 isotype). (+) cells treated with the anti-ROR1 mAb clone 5F1. (S) cells treated with staurosporine.

Western blot analyses for cleaved PARP and caspase-8/9 as well as downregulation of MCL-1 were done using protein lysates prepared from the 24 h apoptosis experiments. The effects of the anti-ROR1 mAb clone 5F1 were tested on the ESTDAB049, ESTDAB112 and A375 melanoma cells. The anti-ROR1 mAbs induced cleavage of PARP, caspase 8 and caspase 9 as well as down-regulation of MCL-1 (Fig. 2D).

Staurosporine was used as a positive control for apoptosis induction. More than 70% of cells had gone into apoptosis after 24 h incubation (data not shown). Staurosporine also induced a significant PARP, caspase 8 and 9 cleavage as well as MCL-1 downregulation (Fig. 2D).

### Cytotoxic effects of anti-ROR1 mAbs in CDC

The effect of anti-ROR1 mAbs in CDC was evaluated after 2 h incubation of cells in the presence of human complement. Anti-ROR1 mAbs could activate complement to lyse melanoma cells to a varying degree. The CDC activity of the various mAbs against the different cell lines are shown in Figure 3A–C. The anti-ROR1 mAb clone 1E9 had the lowest CDC activity against the A375 cell line. Lysis of all mAbs in the presence of complement using the 7 melanoma cell lines (except for anti-ROR1 mAb clone 1E9 on A375 cell line) was statistically significant compared to no complement (p<0.01). No CDC activity was seen using the ROR1 negative T47D cell line (Fig. 3C). Comparison of 4 mAbs in CDC showed a significantly better effect of mAb 5F1 compared to 3H9 using ESTDA049 (p = 0.01), of 3H9 on the ESTDAB075 cell line compared to the other 3 mAbs (p = 0.01-0.001), of mAb 3H9 compared to 5F1 on ESTDAB094 (p = 0.01) and of mAbs 1A8, 5F1 and 3H9 compared to 1E9 mAb on the A375 cell line (p = 0.01-0.0001).

**Figure 3:** Anti-ROR1 mAbs in complement dependent cytotoxicity (CDC). Frequency (%) (mean+SEM) of apoptotic/necrotic cells (Annexin-V^+^/PI^+^) induced by 4 anti-ROR1 mAbs with (▪) or without (□) human complement using various ESTDAB (A, B), DFW and A375 melanoma cell lines (C). The T47D cell line did not express ROR1. ^*^P = 0.01; ^**^P = 0.001. P-values refer to comparison with and without complement for the respective mAbs. NR mAb: non-relevant isotype control mAb (mouse IgG1 isotype), C: Complement.

### Antibody dependent cell-mediated cytotoxicity (ADCC)

Purified NK cells were used as effector cells. Various effects of the anti-ROR1 mAbs were noted (Fig. 4). The lowest and highest cytotoxic activity was observed for the anti-ROR1 mAb clone 5F1 on DFW (Fig. 4A) and ESTDAB081 (Fig. 4B). The effects of the anti-ROR1 mAbs on melanoma cell lines was statistically significant compared to the non-relevant isotype control mAb (mouse IgG1 isotype) as well as in comparison to the ROR1 negative cell line T47D (P = 0.05-0.0001).

**Figure 4:** Cytotoxic effects of anti-ROR1 mAbs in the presence of NK cells (ADCC). Frequency (%) (mean+SEM) of apoptotic/necrotic cells (Annexin-V^+^/PI^+^) induced by 4 anti-ROR1 mAbs and a non-relevant isotype control mAb (mouse IgG1 isotype) in the presence of NK cells at different target: effector ratios. Target cells: ESTDAB049 (□), 075 (), DFW (▪), A375 () (A) and ESTDAB081 (□), 094 (), 112 (▪) melanoma cells and T47D () as a ROR1 negative cell line (B). ADCC of the melanoma cells induced by the anti-ROR1 mAbs compared to the non-relevant isotype control mAb (mouse IgG1 isotype) as wells as to the T47D cell line was statistically significant (P = 0.05-0.0001).

### Silencing of ROR1 in melanoma cells by siRNA

A ROR1 specific siRNA was used to suppress ROR1 expression in those melanoma cell lines that were most sensitive to the direct apoptotic effect of the anti-ROR1 mAbs (ESTDAB049, 075, 112, DFW and A375) as well as the ESTDAB081 melanoma cell line which was resistant to apoptosis by anti-ROR1 mAbs. Transfection of melanoma cells induced a marked decrease in the ROR1 gene-expression (RT-PCR) (Fig. 5A). ROR1 was also downregulated at the protein level (Fig. 5B). Silencing of ROR1 induced apoptosis of the ROR1 positive melanoma cell lines but not of the T47D ROR1 negative cell line (Fig. 6). Morphological changes of the cells typical for apoptosis were noted by light microscopy as well as loss of adherence to tissue culture plates (data not shown).

**Figure 5:** Transfection of melanoma cells (n = 6) using ROR1 suppressing siRNA. Downregulation of ROR1 mRNA (RT-PCR) (A). Downregulation of the ROR1 protein (130 kDa) expression (B). (−) untreated cells, (C) control siRNA treated cells, (+) ROR1 siRNA treated cells.

**Figure 6:** Apoptosis of melanoma cells treated with siROR1. Dot plot (frequency) of apoptotic/necrotic melanoma cells (Annexin-V^+^/PI^+^) treated with siRNA, control siRNA and untreated. Within each quadrant the frequency of apoptotic cells is shown. Results are presented for the ESTDAB049, ESTDAB075, A375, ESTDAB112 (sensitive to apoptosis by anti-ROR1 mAbs) and ESTDAB081 (resistant to apoptosis by anti-ROR1 mAbs), The cell lines T74D cell line was used as a ROR1 negative control.

## Discussion

ROR1 is not only overexpressed in hematologic malignancies, but also in solid tumors [13], [15], [30]–[32]. ROR1 knockdown prevented growth of primary leukemic cells as well as of breast cancer cells in vitro and in vivo [13], [16], [19]. ROR1 was constitutively phosphorylated in CLL and cell lines of different origins [16], [18]. Current evidence suggests that ROR1 might play a role as a survival factor for various malignancies and to be an interesting target for therapy [13], [15], [17], [20].

In the present study we could show that melanoma cell lines expressed a 130 kDa ROR1 protein, corresponding to the fully glycosylated isoform [33]. A proportion of melanoma cell lines did however not express ROR1 on the surface or at least not detectable by our anti-ROR1 mAbs. This subpopulation might represent melanoma cells with a low proliferative activity as ROR1 has been shown to be expressed in less mature cells with a high rate of cell division [15]. ROR1 was phosphorylated at serine and tyrosine residues. Transfection of melanoma cells using ROR1 siRNA, downregulated ROR1, which was proceeded by apoptosis. Specific anti-ROR1 mAbs induced apoptosis of the melanoma cells.

Functional characteristics of cellular proteins are related to post-translational modifications, as glycosylation, forming a unique functional glycan in the tissue [34]–[35]. Aberrant glycosylation has been demonstrated for various proteins in melanoma cells with functional consequences [27]. The ESTDAB series of melanoma cell lines showed different glycan patterns which related to clinical characteristics of the patients from which the cell lines were derived [21], [27]–[29].

Depending on the glycosylation pattern of an antigen, a targeting mAb may induce various effects upon binding [36]. The frequency of ROR1 positive cells did not differ markedly between the various melanoma cell lines, but a significant variation in the cytotoxic effects of the different anti-ROR1 mAbs was noted. The ESTDAB081 cell line was resistant to the apoptotic effect of the anti-ROR1 mAbs, but not to siRNA. These variations might mirror post-translation modifications of ROR1, as well as the epitopes recognized by the mAbs in addition to other factors of importance for drug resistance [36]–[37]. Gene silencing of ROR1 induced apoptosis also in mAb resistant cells indicating that some ROR1 mAbs may not mediate a proper apoptotic signal.

The induction of direct apoptosis of melanoma cells is in agreement with recent findings demonstrating the same phenomenon in primary CLL leukemic cells [18], [20]. Targeting ROR1 in CLL with anti-ROR1 mAbs induced rapid dephosphorylation of ROR1 preceding apoptosis [18], [20]. Mechanisms of action for induction of apoptosis by anti-ROR1 antibodies are not well understood but pathways as AKT/CREB may be involved [18], [20], [31], [38]. The A375 melanoma cell line has been shown to express activated BRAF and mediate a strong BRAF/MEK/ERK signal [39]. Whether ROR1 activation might be associated with the BRAF/MEK/ERK signaling pathway or if blocking of ROR1 may mediate cell death through this pathway is not known.

Phosphorylation of serine and tyrosine residues is important for regulating protein activities including RTKs [40]–[42]. ROR1 as well as ErbB2 are both members of the type I RTK subclass, contributing to the malignant transformation of various human cancers. High expression of HER1/2, VEGFR_2_/KRD and estrogen receptors and their tyrosine phosphorylation in breast cancer correlated with a poor prognosis [40], [43]–[44]. Our findings, showing phosphorylation of ROR1 at tyrosine and serine residues in melanoma cell lines is of interest. We have recently shown that ROR1 is highly phosphorylated in progressive compared to non-progressive CLL [18]. Furthermore, mouse ROR1 is phosphorylated at the serine position 652 located in the activation segment of ROR1 both in the human and mouse ROR1 protein and may be an important site to be triggered by serine/threonine kinases [45]. It is not clear if phosphorylation of ROR1 at tyrosine [46]–[48] or serine [49]–[50] residues is due to autophosphorylation or not. Tyrosine and serine phosphorylation might be triggered by other kinases [51].

Expression of ROR1 has previously been shown in 3 melanoma cell lines including SK-MEL 2, 5 and 28 and ROR1 was phosphorylated at tyrosine and serine residues [16]. SiRNA transfection prevented cell growth only in a low numbers of cells, probably due to a low expression and phosphorylation of ROR1. However, a high degree of growth inhibition was observed in the ROR1 high expressing non-melanoma cell lines NCI-H1993 and HS746T [16]. These two cell lines had an abnormality in the Met oncogene inducing activation of Met. ROR1 might have been phosphorylated by Met as a result of transphosphorylation but a low degree of autophosphorylation could also be seen [16]. To our knowledge, there is no report showing aberrant expression of the Met oncogene in those melanoma cell lines we used. Our data may support the suggestion that the Met RTK is not the only RTK to phosphorylate ROR1 [13], [15]–[16], [31]. Other modifications might contribute to the functional properties of ROR1 [52]–[53]. Furthermore, cells expressing endogenously upregulated ROR1 might be differently activated compared to transfected cells [54]–[55].

In summary, we described for the first time the expression of ROR1 at the mRNA and protein levels in melanoma cells and could show that targeting melanoma cells by anti-ROR1 mAbs and ROR1 suppressing RNA induced apoptosis of the cells. Further studies on the biology of ROR1 in melanoma are warranted as well as to develop anti-ROR1 targeted therapy.
